# Curative Effect of Early Full Nursing Combined with Postdischarge Continuation Nursing on Patients after Craniocerebral Trauma

**DOI:** 10.1155/2021/7424855

**Published:** 2021-09-04

**Authors:** Xiaodan Lv, Fengxia Lv, Guimei Yin, Ju Yi, Yi Liu, Ying Tian

**Affiliations:** ^1^Department II of Neurosurgery, The First Affiliated Hospital of Kunming Medical University, Kunming 650000, Yunnan, China; ^2^Panzhihua Center for Disease Control and Prevention, Panzhihua 617099, Sichuan, China; ^3^Department of Nursing, The First Affiliated Hospital of Kunming Medical University, Kunming 650000, Yunnan, China

## Abstract

Early full nursing helps patients with some dysfunctions speed up the reorganization of central nervous system functions and coordinate muscle and limb activities. Postdischarge continuation nursing for patients who have not fully recovered after being discharged from the hospital can transfer nursing work from the hospital to the family to meet their nursing needs. In this study, early full nursing combined with postdischarge continuation nursing was used for patients with traumatic brain injury to explore its efficacy and its impact on patients' motor function, quality of life, and complications. The results of the study show that the total effective rate of the observation group (95.92%) was higher than that of the control group (85.71%). At discharge and 1 month, 3 months, and 6 months after discharge, the upper limb Fugl-Meyer score, lower limb Fugl-Meyer score, ARAT score, FIM score, 4 dimensions of GQOLI-74 score, and Barthel index scores of the observation group were higher than those of the control group in the same period. The postoperative complication rate (10.20%) of the observation group was lower than that of the control group (26.53%). Early full nursing combined with postdischarge continuation nursing can improve the rehabilitation effect, effectively promote the recovery of motor function in patients with traumatic brain injury, improve the quality of life, and reduce postoperative complications.

## 1. Introduction

Craniocerebral trauma is one of the common emergency departments of brain surgery, and its clinical symptoms are head trauma, hemorrhage, intracranial hypertension and disturbance of consciousness caused by trauma [1, 2]. The brain tissue damage of the patient causes the nervous system function to be affected, which affects the cognitive ability, motor function, and inconvenience to daily life [3, 4]. Early full nursing for some patients with dysfunction is helpful to accelerate the reorganization of central nervous system function and coordinate muscle and limb activities [5, 6]. For patients who have not fully recovered their health after being discharged from the hospital, continuation nursing can transfer nursing work from the hospital to the family to meet their nursing needs [7, 8]. This study explored the effect of early full nursing combined with postdischarge continuation nursing on the motor function, quality of life, and complications of patients after traumatic brain injury. The specific report is as follows.

## 2. Materials and Methods

### 2.1. Patients

We selected 136 patients with craniocerebral trauma admitted to our hospital from May 2018 to December 2019, including 79 males and 57 females, aged 18 to 60 years, average age 38.19 ± 20.44 years old. Causes of injury: 48 patients of falls from heights, 42 patients of traffic accidents, 29 patients of blunt contusion, and 17 patients of other reasons. Injury type: 49 patients of brain contusion, 36 patients of epidural hematoma, 20 patients of intracranial injury, 19 patients of skull fracture, and 12 patients of other types. Inclusion criteria: age ≥18 years, diagnosis of craniocerebral injury by CT or MRI, and expected hospital stay ≥2 weeks. Exclusion criteria: patients with severe heart, lung, kidney, and other organ dysfunction, patients with mental disorders, And patients with other cranial nerve diseases. All patients were divided into the observation group and the control group by a random number table, with 68 patients in each group. During the study, 15 patients in the control group excluded the study due to death, 4 patients gave up continuing treatment, 17 patients in the observation group excluded the study due to death, and 2 patients gave up continuing treatment. In the end, 49 patients of the control group participated in the study, and 49 patients of the observation group participated in the study. The control group included 27 males and 22 females, aged 21 to 60 years, average age 38.82 ± 19.22 years old. Causes of injury: 17 patients of falls from heights, 17 patients of traffic accidents, 9 patients of blunt contusion, and 6 patients of other reasons. Injury type: 17 patients of brain contusion, 11 patients of epidural hematoma, 9 patients of intracranial injury, 8 patients of skull fracture, and 4 patients of other types. The observation group included 29 males and 20 females, aged 19 to 56 years, average age 37.56 ± 18.94 years old. Causes of injury: 16 patients of falls from heights, 15 patients of traffic accidents, 10 patients of blunt contusion, and 8 patients of other reasons. Injury type: 19 patients of brain contusion, 10 patients of epidural hematoma, 8 patients of intracranial injury, 9 patients of skull fracture, and 3 patients of other types. There was no statistically significant difference between the two groups of patients in general information (*P* > 0.05).

### 2.2. Research Method

Both groups of patients underwent corresponding surgical treatment according to their specific injuries. The control group received routine nursing during hospitalization and postdischarge continuation nursing. Routine nursing: emergency rescue, perioperative nursing intervention, postoperative condition observation, etc. Postdischarge continuation nursing: telephone follow-up once per week within 1 month after discharge and 1 telephone follow-up 2 weeks from the second month after discharge. The follow-up includes specific health knowledge, assessment of recovery, supervision of medication, guide for rehabilitation skills and training, and guide for mental health problems.

On the basis of the control group, the observation group implemented early full nursing during the hospitalization. Early full nursing: (1) to conduct a comprehensive assessment of the patient's condition after the operation and teach the patient the concept of rehabilitation training. (2) After the patient's vital signs are stable, timely rehabilitation exercises are carried out, including massage treatments: massaging and rubbing the limbs and feeling irritation. The technique ranges from light to heavy, from slow to fast, once every 4 to 6 h, every 10 min, 3 to 4 times a day, each joint movement 5 to 6 times; attention should be paid to gentle movements to avoid new injuries. Changing position: partial joint activities can be carried out 24 h after trauma or after surgery, such as finger joints, wrist joints, elbow joints, and ankle joints. We should be careful not to use excessive force during activities to prevent new damage to joints, ligaments, and muscles and follow the principle of gradual progress. Joint flexion and extension: including the elevation and flexion and extension activities of the shoulder, elbow, knee, hip, and ankle joints, the activity intensity is subject to the patient's tolerance. The intensity is gradually increased, the extension and flexion are maintained for 10 s and alternated, tightening the thighs is assisted, the toes are straightened for 10 s and then relaxed, and the lower limbs are elevated and gradually transitioned from 30° to 45°–60°. (3) After the patient's condition is basically stable, the patient is instructed to perform balance training, standing training, walking training, and other sports functions, and gradually, the patient's self-care ability is trained such as dressing, washing, and eating. (4) Communication and exchanges are enhanced with patients during exercise, early psychological counseling is patiently performed, patients are actively enlightened, and psychological rehabilitation counseling is provided.

### 2.3. Observation Index

At admission and 6 months after discharge, the two groups of patients were scored on the National Institutes of Health Stroke Scale (NIHSS). The curative effect was evaluated by the decrease of NIHSS score, and the curative effect grade was divided into cure, significant effect, effective, and invalid. Cure : NIHSS score decrease >90%. Significant effect: NIHSS score decrease 46% to 90%. Effective: NIHSS score decrease 18% to 45%. Invalid: NIHSS score decrease ≤17%. Total effective rate = (number of cured + number of significant effect + number of effective)/total number of patients ×100%. At admission and discharge, 1 month, 3 months, and 6 months after discharge, the patients in the two groups were treated with the Fugl-Meyer motor function scale (FMA) and upper limb movement study scale (ARAT), functional independence which refers to the functional independence assessment scale (FIM), comprehensive quality of life assessment questionnaire (Generic Quality of Life Inventory 74, GQOLI-74), and Barthel index scores. The higher the FMA, ARAT, and FIM scores, the better the limb function. GQOLI-74 is divided into four dimensions: physical function, psychological function, social function, and material life. The higher the score, the better the quality of life. The higher the Barthel index score, the better the self-care ability. During the follow-up, postoperative complications were recorded. The flow of experiment is shown in Figure 1.

### 2.4. Statistical Method

The results of this experiment were statistically analyzed by SPSS 20.0 (SPSS Co., Ltd., Chicago, USA). Count data were expressed by (rate), and the chi-square test was used for their comparison between groups. Measurement data were expressed by (mean ± standard deviation), the analysis of variance using repeated measurement design was compared, and the *t*-test was used for their comparison between groups. *P* < 0.05 indicates that the difference is statistically significant.

## 3. Results

### 3.1. Comparison of Clinical Efficacy between the Two Groups

In this study, the control group 12 patients were cured, 23 patients were significant effective, 7 patients were effective, and 7 patients were invalid. In the observation group, 16 patients were cured, 26 patients were significant effective, 5 patients were effective, and 2 patients were invalid. The total effective rate of the observation group, 47 (95.92%), was higher than that of the control group, 42 (85.71%), and the difference was statistically significant (*P* < 0.05), as shown in Figure 2.

### 3.2. Comparison of Motor Function between the Two Groups in Different Periods

At the time of admission, there was no significant difference between the upper limb Fugl-Meyer score, lower limb Fugl-Meyer score, ARAT score, and FIM score between the two groups (*P* > 0.05). At discharge and 1 month, 3 months, and 6 months after discharge, the upper limb Fugl-Meyer score, lower limb Fugl-Meyer score, ARAT score, and FIM score of the two groups were higher than those at admission, and the observation group was higher than the control group in the same period; the difference was statistically significant (*P* < 0.05), as shown in Figure 3.

### 3.3. Comparison of Quality of Life between the Two Groups in Different Periods

At the time of admission, there was no statistical difference in the 4 dimensions of physical function, mental function, social function, and material life in the two groups of GQOLI-74 (*P* > 0.05). At discharge and at 1 month, 3 months, and 6 months after discharge, the scores of 4 dimensions of GQOLI-74 in the two groups were higher than that at admission, and the observation group was higher than the control group at the same time; the differences were statistically significant (*P* < 0.05), as shown in Figure 4.

### 3.4. Comparison of Self-Care Ability Scores between the Two Groups in Different Periods

At the time of admission, there was no significant difference in Barthel index scores between the two groups (*P* > 0.05). At discharge and at 1 month, 3 months, and 6 months after discharge, the Barthel index scores of the two groups were higher than those at admission, and the observation group was higher than the control group at the same time; the difference was statistically significant (*P* < 0.05), as shown in Figure 5.

### 3.5. Comparison of Postoperative Complications between the Two Groups

In the control group, there were 4 patients of dysfunction, 2 patients of memory impairment, 1 patient of brain herniation, 3 patients of infection, and 3 patients of pressure sores. In the observation group, there were 2 patients of dysfunction, 1 patient of memory impairment, 1 patient of infection, and 1 patient of pressure sore. The postoperative complication rate, 5 (10.20%), of the observation group was lower than that of the control group, 13 (26.53%), and the difference was statistically significant (*P* < 0.05), as shown in Figure 6.

## 4. Discussion

Craniocerebral injuries are mainly caused by falls and impacts, which are more common in traffic accidents and construction accidents [9,10]. With the acceleration of social modernization and the rapid development of transportation, construction, and other industries, the incidence of head trauma is gradually increasing [11]. Advances in medical technology have allowed most patients with craniocerebral trauma to receive better treatment. However, due to the damage involving nerve tissues, patients still have different degrees of dysfunction after treatment, such as coma, aphasia, and hemiplegia [12–14]. Therefore, postoperative rehabilitation care is very important for the prognosis of patients with traumatic brain injury.

At the initial stage of brain injury, the structure and function of the central nervous system have the strongest plasticity, which is the best stage for neuron regeneration. Therefore, early rehabilitation training for patients after traumatic brain injury is conducive to the functional reorganization of the nervous system and the recovery of motor functions [15–17]. In this study, the total effective rate of the observation group (95.92%) was significantly higher than the total effective rate of the control group (85.71%), showing that the early full nursing combined with postdischarge continuation nursing has a good recovery effect on patients after traumatic brain injury. This is consistent with the research result of Olson et al. [18]. After craniocerebral injuries, nurses assess patients and develop an understanding of their condition by interpreting the meaning from physiologic and observational or behavioral cues. These interpretations form the basis for optimizing the timing of discrete nursing interventions, the outcome of which influences the trajectory toward recovery or toward secondary brain injury. Early full nursing advocates early rehabilitation exercise for patients. In addition, when patients with craniocerebral trauma are discharged from the hospital, they still have not fully recovered. Postdischarge continuation nursing can help guide patients and their families to learn personal self-care, maintain the patient's condition stable, and improve and restore health [19, 20].

In this study, the four dimensions of the upper limb Fugl-Meyer score, lower limb Fugl-Meyer score, ARAT score, FIM score, and GQOLI-74 scores in the observation group were higher than those of the control group during the same period at different periods after nursing, indicating that the early full nursing combined with postdischarge continuation nursing has a higher effect on improving the motor function and quality of life of patients after craniocerebral trauma. After the patient's vital signs are stable, the concept of rehabilitation training can be taught to the patient and their family members, which can help the patient accept their own condition, correctly understand the development of the disease, and establish a reasonable concept of rehabilitation [21–23]. When the patient's condition tends to be stable, the patient is patiently guided to carry out corresponding rehabilitation exercises around language function, sensory function, motor function, etc., step by step, and gradually restore various nerve and limb functions [24, 25]. Early full nursing should also always pay attention to the patient's mental state. Many patients may experience negative emotions such as depression, disappointment, and collapse due to long-term inability to master physical motor skills. Nurses, caregivers, and family members should promptly persuade and encourage patients to have positive exercise psychology and actively cooperate with the training process [26, 27].

After craniocerebral trauma, the motor function of the limbs is impaired, which leads to a decline in the quality of life. Therefore, it is necessary to restore the patient's limb motor function as soon as possible to improve the patient's self-care ability and quality of life [28]. The results of this study showed that the Barthel index scores of the observation group were significantly better than those of the control group at different periods after nursing. It is suggested that the combination of early full nursing combined with postdischarge continuation nursing can improve the long-term self-care ability and quality of life of patients. Early functional exercise can promote the restoration of physiological functions, reduce the probability of disability, and accelerate the recovery of limb function, which plays a key role in restoring the patient's ability of daily living and quality of life. Postdischarge continuation nursing is based on the characteristics of the patient's postoperative recovery. The rehabilitation process is divided into different stages. Different rehabilitation nursing contents are formulated at different stages, and different rehabilitation nursing plans are completed, following the principle of gradual progress. Patients' confidence in rehabilitation training is effectively improved, the reconstruction of normal functional activities is speeded up, and the maximum recovery of various functions such as sports is achieved [29, 30].

In this study, the incidence of postoperative complications in the observation group (10.20%) was significantly lower than that in the control group (26.53%). Early full nursing combined with postdischarge continuation nursing can reduce complications. Early full nursing develops a rehabilitation plan for the patient, helps the patient to carry out exercise training as soon as possible, and reduces the time in bed to reduce the incidence of infection, bedsores, and other complications.

## 5. Conclusions

This study applies early full nursing combined with postdischarge continuation nursing to patients after craniocerebral trauma. The results show that early full nursing combined with postdischarge continuation nursing can improve the postoperative rehabilitation efficacy of patients and effectively promote the recovery of motor function and self-care after surgery. It has the ability to improve the quality of life of patients and reduce the probability of postoperative complications. However, there are also shortcomings such as small sample size, which requires further multicenter and in-depth research.

## Figures and Tables

**Figure 1:** Experimental flowchart.

**Figure 2:** Comparison of clinical efficacy between the control group and the observation group. Note: compared with the control group, ^*∗*^*P* < 0.05.

**Figure 3:** Comparison of motor function between the control group and the observation group in different periods. Note: compared with the same group, ^*∗*^*P* < 0.05. Compared with the control group in the same period, ^#^*P* < 0.05. Compared with the control group in admission, *P* > 0.05.

**Figure 4:** Comparison of quality of life between the control group and the observation group in different periods. Note: compared with the same group, ^*∗*^*P* < 0.05. Compared with the control group in the same period, ^#^*P* < 0.05. Compared with the control group in admission, *P* > 0.05.

**Figure 5:** Comparison of self-care ability scores between the control group and the observation group in different periods. Note: compared with the same group, ^*∗*^*P* < 0.05. Compared with the control group in the same period, ^#^*P* < 0.05. Compared with the control group in admission, *P* > 0.05.

**Figure 6:** Comparison of postoperative complications between the control group and the observation group. Note: compared with the control group, ^*∗*^*P* < 0.05.

## Data Availability

The analyzed data can be obtained for noncommercial use by contacting the corresponding author.
